The article "Investigation of Three-Dimensional Condensation Film Problem over an Inclined Rotating Disk Using a Nonlinear Autoregressive Exogenous Model" was published in 2022. Journal: Comput Intell Neurosci.

# Investigation of Three-Dimensional Condensation Film Problem over an Inclined Rotating Disk Using a Nonlinear Autoregressive Exogenous Model

**DOI:** 10.1155/2022/2930920

**Published:** 2022-02-10

**Authors:** Naveed Ahmad Khan, Muhammad Sulaiman, Ebenezer Bonyah, Jamel Seidu, Fahad Sameer Alshammari

**Affiliations:** ^1^Department of Mathematics, Abdul Wali Khan University Mardan, Mardan, Khyber Pakhtunkhwa, Pakistan; ^2^Department of Mathematics Education, Akenten Appiah-Menka University of Skills Training and Entrepreneurial Development, Kumasi, Ghana; ^3^School of Railways and Infrastructure Development, University of Mines and Technology (UMaT) Essikado, Sekondi-Takoradi, Ghana; ^4^Department of Mathematics, College of Science and Humanities in Alkharj, Prince Sattam Bin Abdulaziz University, Al-Kharj 11942, Saudi Arabia

## Abstract

This paper analyzed the three-dimensional (3D) condensation film problem over an inclined rotating disk. The mathematical model of the problem is governed by nonlinear partial differential equations (NPDE's), which are reduced to the system of nonlinear ordinary differential equations (NODE's) using a similarity transformation. Furthermore, the system of NODEs is solved by the supervised machine learning strategy of the nonlinear autoregressive exogenous (NARX) neural network model with the Levenberg–Marquardt algorithm. The dimensionless profiles of velocity, acceleration, and temperature are investigated under the effect of variations in the Prandtl number and normalized thickness of the film. The results demonstrate that increasing the Prandtl number causes an increase in the fluid's temperature profile. The solutions obtained by the proposed algorithm are compared with the state-of-the-art techniques that show the accuracy of the approximate solutions by NARX-BLM. The mean percentage errors in the results by the proposed algorithm for Θ(*η*), Ψ(*η*), *k*(*η*), −*s*(*η*), and (*θ*(*η*)) are 0.0000180%, 0.000084%, 0.0000135%, 0.000075%, and 0.00026%, respectively. The values of performance indicators, such as mean square error and absolute errors, are approaching zero. Thus, it validates the worth and efficiency of the design scheme.

## 1. Introduction

The liquid condensate removal from cooled, saturated vapors is of immense significance in various domains of engineering, such as coating and cooling with spray, and the mechanisms of chemical vapor accumulation are widely used in the production of thin film in semiconductor industries. Many researchers have conducted a well-known study to investigate the physical model and heat transfer of the fluid with different conditions. Nusselt [1], in 1916, studied the condensation over a vertical plate that formed the basis for many researchers to study the condensation of different fluid problems. Nusselt's solution was developed by Koh et al. [2] under the consideration of convective terms, inertia, and vapor resistance in the condensation of fluid flow. The condensation of the rotating disk in steady vapor with a large volume is studied by Sparrow et al. [3]. They extended the idea of Karman V. [4] on the rotating disk, in which the Navier–Stokes equations are transformed into the set of nonlinear ordinary differential equations (NODE's) and solved numerically for the solutions corresponding to different values of finite film thickness. Becket et al. [5] and Chary and Sarma [6] further broadened the work of Nusselt by adding vapor drag and suction on the plate.

The article "Investigation of Three-Dimensional Condensation Film Problem over an Inclined Rotating Disk Using a Nonlinear Autoregressive Exogenous Model" was published in 2022. Journal: Comput Intell Neurosci.

The flow of a liquid film is made of condensing liquid on a disc and is nonlinear in nature. Generally, finding the exact and analytical solutions to such a problem is a difficult task. Different researchers have adopted various methods to find a solution for the three-dimensional condensation film problem. The governing model of the 3D flow of fluid is transformed into a set of nonlinear differential equations by Wang C. Y. [7] using the similarity transformation and solving the problem using the perturbation method. Several other techniques are used to solve the condensation film problem, such as homotopy analysis method (HAM) [8], homotopy perturbation method (HAM) [9, 10], classical Runge–Kutta and shooting method [11], extended optimal homotopy asymptotic method (EOHAM) [12], variational iteration method (VIM) [13], control volume finite element method (CVFEM) [14], differential transformation method (DTM) [15], spectral quasi linearization method (SQLM) [16], optimal homotopy analysis method (OHAM) [17], variation of parameter method (VPM) [18], and Akbari-Ganji method (AGM) [19].

In this paper, a liquid film created by the condensing fluid on a revolving disc under the centrifugal and gravitational forces is considered. A supervised learning technique is proposed to solve the system of NODE's effectively. The classical numerical approaches mostly convert the governing equations comprising partial differential equations into a discretized model that appears in the form of a set of algebraic linear or nonlinear equations. To solve a set of algebraic equations, considerable computational time and memory requirements are needed by direct solvers. In addition, such techniques are gradient-based methods with deterministic approaches. To overcome these drawbacks, artificial intelligence-based supervised learning techniques are designed that are free of gradient and only require the essential initial parameter and terminal conditions for execution. Some recent applications of the stochastic techniques include the solutions for the saturation of water and oil [20], absorption of carbon dioxide [21], the corneal model for eye surgery [22], and the temperature distribution of conductive-convective and radiative fins [23]. These facts inspire authors to explore and incorporate the intelligent strength of artificial neural networks to solve the problem formed by the condensation of 3D-fluid flow on a rotating disk. The novel contributions of the presented study are summarized as follows:

- The problem of a three-dimensional (3D) condensation layer over an inclined rotating disc is investigated in this article. The governing mathematical model of the problem is given by nonlinear partial differential equations (PDE's), which are transformed into the set of nonlinear ordinary differential equations (ODE's) using similarity transformations.
- The dimensionless profiles of velocity, acceleration, and temperature of the problem are investigated under the effect of variations in the Prandtl number and normalized thickness by developing a supervised machine learning strategy using NARX neural networks with the backpropagated Levenberg–Marquardt algorithm.
- The accuracy of the results obtained by the design algorithm is measured by comparison with the state-of-the-art techniques.
- The results of mean percentage errors and performance indicators in terms of mean square error (RMSE), mean absolute deviations (MAD), absolute errors (AE), error in Nash Sutcliffe efficiency (ENSE), and Theil's inequality coefficient (TIC) are defined to validate the worth and accuracy of the design algorithm.

The article "Investigation of Three-Dimensional Condensation Film Problem over an Inclined Rotating Disk Using a Nonlinear Autoregressive Exogenous Model" was published in 2022. Journal: Comput Intell Neurosci.

## 2. Problem Formulation

Figure 1 illustrates the rotating disk with an angular velocity Ω that is inclined at an angle *β* with a horizontal axis. A film of fluid with thickness *t* is formed by spraying on the disk with a velocity *W*. It is assumed that the film thickness is negligible as compared to the radius of the disk, and therefore, the end effects are ignored. $T_{\bar{w}}$ and *T*_0_ denote the temperatures on the disk and film surface, respectively. The ambient pressure (*p*_0_) on the film surface is assumed to be the function of *z*. The problem is expressed mathematically in the coordinate system (*x*, *y*, *z*), with the *z* axis being the rotation axis. The continuity, momentum, and energy equation after neglecting the viscous dissipation can be written as [7, 8] follows:

(1) $$\begin{array}{c} U_{x}+U_{y}+U_{z}=0, \end{array}$$

(2) $$\begin{array}{c} UU_{x}+VU_{y}+\bar{w}U_{z}-g\;\sin\;\beta =\vartheta \left(U_{xx}+U_{yy}+U_{zz}\right), \end{array}$$

(3) $$\begin{array}{c} UV_{x}+VV_{y}+\bar{w}V_{z}=\vartheta \left(V_{xx}+V_{yy}+V_{zz}\right), \end{array}$$

(4) $$\begin{array}{c} U{\bar{w}}_{x}+V{\bar{w}}_{y}+\bar{w}{\bar{w}}_{z}-\vartheta \left({\bar{w}}_{xx}+{\bar{w}}_{yy}+{\bar{w}}_{zz}\right)+g\;\cos\;\beta =-\frac{P_{z}}{\rho }, \end{array}$$

(5) $$\begin{array}{c} UT_{x}+VT_{y}+\bar{w}T_{z}=\alpha \left(T_{xx}+T_{yy}+T_{zz}\right), \end{array}$$

*U*, *V*, and $\bar{w}$ are the components of velocity in *x*, *y*, and *z* directions. *T* is the temperature. *α*, *ρ*, and *ϑ* are the thermal diffusion, density, and kinematic viscosity of the fluid. For boundary conditions, zero shear stress on the surface of the film and zero slip on the disk are assumed. Thus, the boundary conditions (B.C) are given as follows:

(6) $$\begin{array}{c} T=T_{w},\\ U=-\Omega y,\\ \bar{w}=0,\\ V=\Omega x,\;\text{at }z=0\\ p=p_{0},\\ U_{z}=0,\\ \bar{w}=-W,\\ V_{z}=0,\\ T=T_{0},\;\text{at }z=t. \end{array}$$

In 2007, Wang C. Y. [7] introduced a transformation for the abovementioned problem, which is as follows:

(7) $$\begin{array}{c} U-\psi k\left(\eta \right)\sin\frac{\beta }{\Omega }=-\Omega y\Psi \left(\eta \right)+\Omega x\Theta^{\prime }\left(\eta \right),\\ V-gs\left(\eta \right)\sin\frac{\beta }{\Omega }=\Omega x\Psi \left(\eta \right)+\Omega y\Theta^{\prime }\left(\eta \right),\\ \bar{w}+2\sqrt{\Omega }\vartheta \Theta \left(\eta \right)=0,\\ T-T_{\bar{w}}=\left(T_{0}-T_{\bar{w}}\right)\theta \left(\eta \right), \end{array}$$

where *η* is defined as

(8) $$\begin{array}{c} \eta =z\sqrt{\frac{\Omega }{\vartheta }}, \end{array}$$

and (1) is satisfied identically using the above transformation in (2) and (4), which can be written as

(9) $$\begin{array}{c} \Theta^{\prime \prime \prime }-{\left(\Theta^{\prime }\right)}^{2}+\Psi^{2}+2\Theta \Theta^{\prime \prime }=0, \end{array}$$

(10) $$\begin{array}{c} \psi^{\prime \prime }-2\Psi \Theta^{\prime }+2\Theta \Psi^{\prime }=0, \end{array}$$

(11) $$\begin{array}{c} k^{\prime \prime }-k\Theta^{\prime }+s\Psi +2\Theta k^{\prime }+1=0, \end{array}$$

(12) $$\begin{array}{c} s^{\prime \prime }-k\Psi -s\Theta^{\prime }+2\Theta s^{\prime }=0. \end{array}$$

Temperature (*θ*) is assumed as a function of *z* alone, and therefore, (5) can be written as

(13) $$\begin{array}{c} \theta^{\prime \prime }+2\text{Pr}\Theta \theta^{\prime }=0, \end{array}$$

where Pr=*ϑ*/*α* is the Prandtl number. Boundary conditions for equations (9)–(13) are defined as follows:

(14) $$\begin{array}{c} \Theta \left(0\right)=0,\\ \Theta^{\prime }\left(0\right)=0,\\ \Theta^{\prime \prime }\left(\delta \right)=0,\\ \Psi \left(0\right)=1,\\ \Psi^{\prime }\left(\delta \right)=0,\\ k\left(0\right)=0,\\ k^{\prime }\left(\delta \right)=0,\\ s\left(0\right)=0,\\ s^{\prime }\left(\delta \right)=0,\\ \theta \left(0\right)=0,\\ \theta \left(\delta \right)=1, \end{array}$$

where $\delta =t\sqrt{\Omega /\vartheta }$ is the normalized thickness, which is also defined using the spraying velocity or condensation as,

(15) $$\begin{array}{c} \Theta \left(\delta \right)=\frac{W}{2\sqrt{\Omega \vartheta }}\\ =\alpha . \end{array}$$

After the flow field is found, various quantities of the fluid flow can be measured. Integrating (4) will result in the desired equation for pressure distribution of the fluid, which is given as follows:

(16) $$\begin{array}{c} p\left(z\right)=p_{0}-\rho \left\{V\left[{\frac{\partial \bar{w}}{\partial z}|}_{z=t}-\frac{\partial \bar{w}}{\partial z}\right]+\frac{1}{2}\left[{\bar{w}}^{2}\left(t\right)-{\bar{w}}^{2}\left(z\right)\right]-g\;\cos\;\beta \left(z-t\right)\right\}. \end{array}$$

If the force on the net area along *x* and *y* directions are normalized by $g\rho \sqrt{\vartheta /\Omega }\sin\;\beta$, then it is equal to the values of *k*′(0) and *s*′(0), respectively.

The article "Investigation of Three-Dimensional Condensation Film Problem over an Inclined Rotating Disk Using a Nonlinear Autoregressive Exogenous Model" was published in 2022. Journal: Comput Intell Neurosci.

## 3. Design Methodology

### 3.1. Artificial Neural Networks and NARX Model

Before the 1980s, the linear parametric autoregressive (AR), the moving average (MA), and the autoregressive moving average (ARMA) were the most common approaches used by researchers to handle different types of problems [24]. These models were linear and could not be used to forecast nonlinear time-series problems. In addition, artificial neural networks (ANNs) have attracted a lot of attention because of their nonlinear and nonparametric characteristics. ANN's models are adaptive approaches based on data that can learn a system's nonlinear behavior from its historical data without having any prior knowledge of the problem. They are universal approximators for functions. Some recent applications of ANN can be found in [25]. The above-mentioned articles motivate the authors to extend the idea of ANNs to solve a nonlinear problem arising in various fields. The NARX model is a nonlinear version of the autoregressive exogenous (ARX) model that has been widely used in various applications and for modeling a variety of nonlinear dynamical systems. The NARX model is a time-series prediction model based on artificial neural networks. It learns a system's behavior more effectively than other NN's (i.e., the learning gradient method in NARX is superior). Compared to other neural networks, it converges much faster and generalizes the solutions in a much better way [26].

The multilayered perceptron (MLP) architecture underpins the NARX model [27] because of its versatility and simplicity. It is one of the most widely utilized ANN models. Input, hidden, and output layers are present in the MLP and NARX models, however, the NARX model includes the time history of the output signal as one of the inputs. The present input signal and its time history serve as the model's other inputs. The number of output neurons and variables in the problem is equal. Let *h*(·) be a nonlinear mapping function of NARX. It relates the input and output of the system by (17),

(17) $$\begin{array}{c} Y\left[x\right]=h\left(y\left[x-1\right],\ldots ,y\left[x-x_{y}\right],u\left[x-1\right],\ldots ,u\left[x-x_{u}\right]\right)+e\left[x\right], \end{array}$$

*u*[*x*] and *Y*[*x*] represent the input and output of a system. *x*_*u*_ and *x*_*y*_ are the maximum lags for input and output, respectively. *e*[*x*] is a noise or prediction error.

The article "Investigation of Three-Dimensional Condensation Film Problem over an Inclined Rotating Disk Using a Nonlinear Autoregressive Exogenous Model" was published in 2022. Journal: Comput Intell Neurosci.

### 3.2. Learning Strategy and Performance Measures

Based on the representation of the NARX neural network model by equation (17), a data set of inputs and outputs are presented to the model during the training phase. A reference solution of 1001 points for the different cases of the 3D condensation film problem is generated using the Runge–Kutta method (RK-4) with the “NDSolve” package in mathematica. After that, an MLP is created with “nntool” in MATLAB using multiple layers of interconnected neurons with one or more hidden layers and nodes, which are connected in a feed-forward manner between the input and output layers, as shown in Figure 2. The predicted output of the multilayered perceptron is given as

(18) $$\begin{array}{c} {\hat{y}}_{\text{MLP}}=f_{2}\left(W_{2}^{T}f_{1}\left(\eta \right)+b_{2}\right),\\ N=W_{1}^{T}\left(u\right)+b_{1}, \end{array}$$

*u* is the input element of a model, *b*_1_ and *b*_2_ are biased terms in the hidden and output layers. *W*_1_ and *W*_2_ represent the synaptic weights that connect the input to the hidden and the hidden to the output layers. *f*_1_ and *f*_2_ represent the activation functions. In this study, the Log-Sigmoid activation function is used for neurons in the input and output layers. Once the number of weights is determined, a conventional training algorithm, such as the backpropagated Levenberg–Marquardt (BLM) algorithm, can be directly applied. To avoid the overfitting of data during the training phase, 15% of the data is reserved for cross-validation and testing. The flow chart of the problem and working strategy of the NARX-BLM algorithm is shown in Figure 3.

To examine the accuracy and effectiveness of the results obtained by the NARX-BLM algorithm for the 3D condensation film problem, performance indices are defined in terms of mean square error (MSE), mean absolute deviations (MAD), absolute errors (AE), root mean square error (RMSE), error in Nash Sutcliffe efficiency (ENSE), and Theil's inequality coefficient (TIC). Mathematical forms of these indices are given as follows:

(19) $$\begin{array}{c} \text{MSE}=\frac{1}{k}\sum_{j=1}^{k}{\left(\theta_{j}\left(t\right)-{\hat{\theta }}_{j}\left(t\right)\right)}^{2},\\ \text{AE}=\left|\theta_{j}\left(t\right)-{\bar{\theta }}_{j}\left(t\right)\right|,\\ \text{MAD}=\frac{1}{k}\sum_{j=1}^{k}\left|\theta_{j}\left(t\right)-{\bar{\theta }}_{j}\left(t\right)\right|,\\ \text{TIC}=\frac{\sqrt{\left(1/k\right)\sum_{j=1}^{k}{\left(\theta_{j}\left(t\right)-{\hat{\theta }}_{j}\right)}^{2}}}{\sqrt{\left(1/k\right)\sum_{j=1}^{k}{\left(\theta_{j}\left(t\right)\right)}^{2}}+\sqrt{\left(1/k\right)\sum_{j=1}^{k}{\left({\hat{\theta }}_{j}\right)}^{2}}}\\ \text{ NSE}=\left\{1-\frac{\sum_{j=1}^{k}{\left(\theta_{j}\left(t\right)-{\bar{\theta }}_{j}\left(t\right)\right)}^{2}}{\sum_{j=1}^{k}{\left(\theta_{j}\left(t\right)-{\hat{\theta }}_{j}\left(t\right)\right)}^{2}},\;\hat{\theta }\left(x\right)=\frac{1}{k}\sum_{j=1}^{k}\theta_{j}\left(t\right),\right.\\ \text{ENSE}=1-\text{NSE}, \end{array}$$

where ${\bar{\theta }}_{j}$, *θ*_*j*_, and ${\hat{\theta }}_{j}$ denote the approximate, reference, and mean solution at *j* th input. *k* denotes the number of grid points. For perfect modeling of the solutions, the desired values of AE, MAD, MSE, RMSE, and ENSE are equal to zero, while the value NSE is one.

The article "Investigation of Three-Dimensional Condensation Film Problem over an Inclined Rotating Disk Using a Nonlinear Autoregressive Exogenous Model" was published in 2022. Journal: Comput Intell Neurosci.

## 4. Numerical Experimentation and Discussion

In this section, an artificial intelligence-based machine leaning algorithm is implemented to study the dimensionless profiles of velocity, acceleration, and temperature of the 3D condensation film problem with an inclined rotating disk under the effect of variations in the Prandtl number and Normalized thickness.

Approximate solutions obtained by the proposed technique for the displacement and velocity profiles of the liquid are shown in Figure 4.  Table 1 shows the comparison of the exact solutions with approximate solutions for Θ, Ψ, *k*, −*s*, and *θ*.  Table 2 shows that the results obtained by the NARX-BLM algorithm overlaps the exact and Akbari–Ganji method solutions with minimum absolute errors (AE) that lie around 3.58 × 10^−05^ to 1.018 × 10^−08^, 1.368 × 10^−05^ to 1.938 × 10^−09^, 1.848 × 10^−04^ to 2.708 × 10^−08^, 1.22 × 10^−05^ to 9.868 × 10^−10^, and 4.23 × 10^−04^ to 4.23 × 10^−09^. The mean percentage error in the approximate solutions by the NARX-BLM algorithm are 0.0000180%, 0.000084%, 0.0000135%, 0.000075%, respectively. These facts demonstrates the accuracy of the solutions when compared with state-of-the-art techniques, such as homotopy perturbation method [9], differential transformation method (DTM) [15], and Akbari–Ganji's method [19]. The sensitivity analysis of the design algorithm in terms of different activation functions (Log-Sigmoid and Tangent Hyperbolic) and for different number of hidden neurons (*n*) in the NARX structure are shown in Tables 3 and 4. The results show that the convergence speed of solutions with Log-sigmoid is much higher than other activation functions.

The article "Investigation of Three-Dimensional Condensation Film Problem over an Inclined Rotating Disk Using a Nonlinear Autoregressive Exogenous Model" was published in 2022. Journal: Comput Intell Neurosci.

Effect of variations in the Prandtl number on the temperature profile of the fluid are illustrated in Figure 5(a). It can be seen that the normalized temperature profile (*θ*(*η*)) for different liquid metals starting from sodium, water, and other higher fluids increases with an increase in the Prandtl number Pr.  Figure 5(b) illustrates the normalized shear stress along the *x* and *y* axis with different normalized film thickness *δ*. When film thickness increases, *k*′(0) increases linearly with high intensity than −*s*′(0).  Figure 6(a) shows the results of Θ^″^(0) and Ψ^″^(0) against *δ*. The results shows that Θ^″^(0) has a maximum value of 0.7085 at *δ*=1.08 and asymptotic to the value at 0.51023. In addition, Ψ(0) possesses a minimum value at *δ*=2.82 and asymptotic to the value at *δ*=6.2.

Furthermore, to validate the efficiency, accuracy, and robustness of the proposed technique, the NARX-BLM algorithm is executed for multiple runs. The results of the mean absolute deviations (MAD), root mean square error (RMSE), Theil's inequality coefficient (TIC), and error in Nash Sutcliffe efficiency (ENSE) in terms of minimum (min), mean, and standard deviations (std.) with different activation functions and the number of neuron architecture of NARX are given in Table 5. The minimum value of MAD, ENSE, RMSE, and TIC with Log-Sigmoid function for Θ(*η*), Ψ(*η*), *k*(*η*), −*s*(*η*), and *θ*(*η*) lies around 10^−5^ to 10^−6^, 10^−12^ to 10^−16^, 10^−4^ to 10^−6^, 10^−5^ to 10^−6^, and 10^−6^ to 10^−8^, respectively. The results of the mean square error and gradient for solutions in equations (9)–(13) are given in Table 6. It can be seen that the results obtained with log-sigmoid activation function are more accurate than the tan-hyperbolic function. The value of MSE for each function lies around 10^−10^ to 10^−15^ as shown in Figure 7.

## 5. Conclusion

The important outcomes of this study are summarized as follows:

- In this paper, we have analyzed the mathematical model of a three-dimensional (3D) condensation film problem over an inclined rotating disk by incorporating the computational strength of the supervised learning method NARX-BLM.
- The designed algorithm is exploited to calculate the numerical solutions for the film problem under the influence of variations in the Prandtl number and normalized thickness.
- The results demonstrate that the increase in the Prandtl number causes an increase in the temperature profile of the film. In addition, *k*′(0) increases linearly with high intensity than −*s*′(0) when the film thickness increases.
- The results obtained by the design algorithm are compared with state-of-the-art techniques, such as the Runge–Kutta method (RK-4), homotopy perturbation method, differential transformation method (DTM), and Akbari–Ganji's method. The statistics of mean percentage error in solutions by the NARX-BLM algorithm establishes the accuracy of the design algorithm.
- Extensive graphical, statistical, and sensitivity analyses are conducted based on performance measures, such as MAD, ENSE, TIC, RMSE, and MSE, which show that the design algorithm is smooth, easy, and efficient for calculating the solutions to real-world problems.

The article "Investigation of Three-Dimensional Condensation Film Problem over an Inclined Rotating Disk Using a Nonlinear Autoregressive Exogenous Model" was published in 2022. Journal: Comput Intell Neurosci.

## Figures and Tables

**Figure 1:** Geometric interpretation of condensation film problem over an inclined rotating disk.

**Figure 2:** Details of a neuron in MLP network.

**Figure 3:** Governing equations of 3D condensation film problem, the NARX model, and working procedure of the proposed algorithm.

**Figure 4:** The change of nondimensional radial velocity and temperature profiles for condensation film problem over an inclined rotating disk with Pr=0.7 and *δ*=1.0.

**Figure 5:** (a) Effect of Prandtl number on the temperature profile of the fluid. (b) Illustrates the normalized shear stress along *x* and *y* axis with different values of normalized film thickness *δ* and Pr=0.7.

**Figure 6:** (a) Influence of changes in the thickness of film on Θ′(0) and Ψ′(0). (b) The results of temperature gradient *θ*′(0) on the disk obtained by the design algorithm with Pr=0.7 against *δ*.

**Figure 7:** Mean values of performance function in term of mean square error and gradient values for condensation film problem over an inclined rotating disk with Pr=0.7 and *δ*=1.0.

**Table 1:** Comparison of solutions obtained by the NARX-BLM algorithm with RK-4 method for Pr=0.7 and *δ*=0.5.

	Θ(*η*)		Ψ(*η*)		*k*(*η*)		−*s*(*η*)		*θ*(*η*)	
*η*	Exact	NARX-BLM	Exact	NARX-BLM	Exact	NARX-BLM	Exact	NARX-BLM	Exact	NARX-BLM
0.00	0	0.000001	1	0.999993	0	0.000340	0	0.000073	0	0.000320
0.05	0.000582	0.000582	0.996086	0.996086	0.023457	0.023457	0.001995	0.001995	0.100279	0.100279
0.10	0.002247	0.002247	0.992286	0.992286	0.044418	0.044418	0.003932	0.003932	0.200554	0.200554
0.15	0.004869	0.004869	0.988700	0.988700	0.062890	0.062890	0.005760	0.005760	0.300813	0.300813
0.20	0.008328	0.008328	0.985417	0.985417	0.078877	0.078877	0.007431	0.007431	0.401036	0.401036
0.25	0.012500	0.012500	0.982514	0.982514	0.092385	0.092385	0.008910	0.008910	0.501201	0.501201
0.30	0.017266	0.017266	0.980055	0.980055	0.103421	0.103421	0.010163	0.010163	0.601278	0.601278
0.35	0.022505	0.022505	0.978090	0.978090	0.111991	0.111991	0.011163	0.011163	0.701234	0.701234
0.40	0.028099	0.028098	0.976660	0.976660	0.118102	0.118102	0.011891	0.011891	0.801032	0.801032
0.45	0.033927	0.033927	0.975792	0.975792	0.121762	0.121762	0.012333	0.012333	0.900634	0.900634
0.50	0.039873	0.039867	0.975501	0.975505	0.122980	0.122980	0.012481	0.012481	1	1

The article "Investigation of Three-Dimensional Condensation Film Problem over an Inclined Rotating Disk Using a Nonlinear Autoregressive Exogenous Model" was published in 2022. Journal: Comput Intell Neurosci.

**Table 2:** Comparison of absolute errors in the solutions of the NARX-BLM algorithm and AG method for Pr=0.7 and *δ*=0.5.

	Θ(*η*)		Ψ(*η*)		*k*(*η*)		−*s*(*η*)		*θ*(*η*)	
*η*	AGM	NARX-BLM	AGM	NARX-BLM	AGM	NARX-BLM	AGM	NARX-BLM	AGM	NARX-BLM
0.00	**0**	1.45*E* − 06	0	1.36*E* − 05	0	1.86*E* − 04	0	1.22*E* − 05	0	6.59*E* − 04
0.05	8.39*E* − 04	**2.57E − 07**	1.06*E* − 06	**8.14E − 08**	6.61*E* − 06	**2.51E − 07**	1.99*E* − 04	**1.32E − 08**	3.40*E* − 05	**8.63E − 07**
0.10	1.43*E* − 04	**1.27E − 07**	5.70*E* − 07	**4.11E − 08**	8.13*E* − 06	**6.75E − 08**	8.32*E* − 05	**2.52E − 08**	5.20*E* − 06	**1.51E − 07**
0.15	7.13*E* − 05	**6.36E − 08**	4.44*E* − 07	**1.11E − 08**	9.26*E* − 06	**2.70E − 08**	6.74*E* − 05	**1.57E − 08**	1.80*E* − 07	**8.76E − 09**
0.20	7.77*E* − 05	**9.79E − 08**	7.10*E* − 07	**9.70E − 09**	1.09*E* − 05	**6.04E − 08**	8.21*E* − 05	**9.86E − 10**	6.47*E* − 07	**2.69E − 07**
0.25	7.01*E* − 05	**1.59E − 08**	7.27*E* − 07	**1.93E − 09**	1.28*E* − 05	**8.26E − 08**	8.61*E* − 05	**1.59E − 08**	5.23*E* − 07	**2.10E − 07**
0.30	6.84*E* − 05	**1.03E − 07**	8.35*E* − 07	**2.95E − 09**	1.48*E* − 05	**4.77E − 08**	9.52*E* − 05	**4.60E − 09**	6.53*E* − 07	**3.91E − 08**
0.35	7.20*E* − 05	**1.01E − 08**	1.00*E* − 06	**1.09E − 08**	1.75*E* − 05	**7.38E − 08**	1.09*E* − 04	**1.46E − 08**	1.80*E* − 07	**2.89E − 07**
0.40	6.32*E* − 05	**1.24E − 07**	7.52*E* − 07	**1.56E − 08**	1.98*E* − 05	**9.77E − 08**	1.09*E* − 04	**2.19E − 08**	1.61*E* − 06	**2.85E − 07**
0.45	4.77*E* − 05	**4.97E − 07**	1.68*E* − 07	**6.17E − 08**	2.09*E* − 05	**2.42E − 07**	9.93*E* − 05	**6.84E − 09**	4.16*E* − 06	**4.96E − 08**
0.50	6.99*E* − 05	**3.58E − 05**	1.09*E* − 06	**4.20E − 07**	2.57*E* − 05	**1.85E − 06**	1.36*E* − 04	**3.65E − 07**	2.52*E* − 08	4.23E − 04

**Table 3:** Sensitivity analysis in terms of AE obtained by the proposed algorithm with different activation functions and neurons in the NARX structure for the condensation film problem with Pr=0.7 and *δ*=1.

	Θ(*η*)				Θ′(*η*)				Ψ(*η*)			
*η*	Log-sigmoid		Tan-sigmoid		Log-sigmoid		Tan-sigmoid		Log-sigmoid		Tan-sigmoid	
	*n* = 60	*n* = 30	*n* = 60	*n* = 30	*n* = 60	*n* = 30	*n* = 60	*n* = 30	*n* = 60	*n* = 30	*n* = 60	*n* = 30
0.0	1.17*E* − 06	3.80*E* − 07	6.09*E* − 07	3.56*E* − 06	1.24*E* − 04	8.82*E* − 05	1.26*E* − 04	1.19*E* − 04	6.83*E* − 06	1.33*E* − 05	1.52*E* − 05	1.15*E* − 05
0.1	7.51*E* − 08	1.14*E* − 08	7.76*E* − 08	1.43*E* − 07	3.11*E* − 07	9.05*E* − 07	1.10*E* − 06	7.27*E* − 07	1.62*E* − 08	8.95*E* − 08	5.04*E* − 08	4.31*E* − 08
0.2	6.19*E* − 08	1.43*E* − 08	4.94*E* − 08	1.28*E* − 08	1.49*E* − 07	1.92*E* − 07	4.21*E* − 07	4.62*E* − 07	3.41*E* − 08	3.49*E* − 08	6.04*E* − 08	3.26*E* − 08
0.3	6.34*E* − 08	3.58*E* − 09	8.48*E* − 09	2.93*E* − 07	1.02*E* − 07	2.35*E* − 07	2.23*E* − 07	9.84*E* − 08	1.23*E* − 09	1.99*E* − 08	3.78*E* − 08	8.42*E* − 09
0.4	7.02*E* − 08	1.01*E* − 08	1.17*E* − 08	2.70*E* − 07	3.75*E* − 08	2.50*E* − 07	1.71*E* − 08	4.16*E* − 08	1.38*E* − 09	8.82*E* − 09	7.22*E* − 09	4.00*E* − 09
0.5	7.57*E* − 08	9.68*E* − 09	2.57*E* − 08	2.00*E* − 07	8.89*E* − 08	1.82*E* − 07	2.17*E* − 08	3.50*E* − 07	5.61*E* − 09	1.37*E* − 08	6.12*E* − 09	1.57*E* − 08
0.6	3.20*E* − 08	4.58*E* − 09	1.54*E* − 08	1.82*E* − 07	4.79*E* − 08	1.46*E* − 07	1.45*E* − 08	3.71*E* − 08	1.61*E* − 08	1.72*E* − 08	7.33*E* − 09	1.69*E* − 08
0.7	1.42*E* − 08	1.51*E* − 08	3.06*E* − 08	3.24*E* − 08	7.27*E* − 08	1.38*E* − 07	1.13*E* − 07	3.68*E* − 07	9.91*E* − 09	1.65*E* − 08	2.86*E* − 09	2.34*E* − 08
0.8	1.97*E* − 07	1.37*E* − 08	7.04*E* − 09	6.92*E* − 07	1.53*E* − 08	2.65*E* − 08	1.63*E* − 07	6.90*E* − 08	2.78*E* − 08	3.20*E* − 08	2.06*E* − 08	1.34*E* − 08
0.9	2.91*E* − 07	7.86*E* − 09	1.02*E* − 07	3.01*E* − 07	1.15*E* − 07	2.09*E* − 07	3.27*E* − 07	2.78*E* − 07	3.95*E* − 08	5.45*E* − 08	6.55*E* − 08	2.72*E* − 08
1.0	2.87*E* − 05	2.37*E* − 05	4.37*E* − 05	6.97*E* − 05	3.68*E* − 06	3.15*E* − 06	4.29*E* − 06	3.36*E* − 06	2.76*E* − 07	4.04*E* − 07	5.65*E* − 07	3.37*E* − 07

The article "Investigation of Three-Dimensional Condensation Film Problem over an Inclined Rotating Disk Using a Nonlinear Autoregressive Exogenous Model" was published in 2022. Journal: Comput Intell Neurosci.

**Table 4:** Sensitivity analysis in terms of AE obtained by the proposed algorithm with different activation functions and neurons in the NARX structure for *k*(*η*), −*s*(*η*), and *θ*(*η*) of the condensation film problem with Pr=0.7 and *δ*=1.

	*k*(*η*)				−*s*(*η*)				*θ*(*η*)			
*η*	Log-sigmoid		Tan-sigmoid		Log-sigmoid		Tan-sigmoid		Log-sigmoid		Tan-sigmoid	
	*n* = 60	*n* = 30	*n* = 60	*n* = 30	*n* = 60	*n* = 30	*n* = 60	*n* = 30	*n* = 60	*n* = 30	*n* = 60	*n* = 30
0.0	9.79*E* − 05	8.97*E* − 05	2.28*E* − 04	1.60*E* − 04	3.71*E* − 05	1.47*E* − 04	1.65*E* − 04	1.49*E* − 04	5.08*E* − 04	8.39*E* − 04	9.72*E* − 04	2.51*E* − 03
0.1	6.46*E* − 08	7.49*E* − 07	3.68*E* − 07	1.46*E* − 07	2.16*E* − 07	2.21*E* − 07	1.33*E* − 06	2.34*E* − 06	3.29*E* − 06	8.38*E* − 06	7.99*E* − 06	2.28*E* − 05
0.2	4.94*E* − 08	8.50*E* − 08	5.65*E* − 07	4.80*E* − 08	2.25*E* − 07	6.00*E* − 07	6.03*E* − 08	2.51*E* − 07	1.34*E* − 06	2.86*E* − 06	2.63*E* − 06	1.83*E* − 05
0.3	3.00*E* − 08	2.73*E* − 07	1.79*E* − 07	4.35*E* − 09	2.23*E* − 07	7.59*E* − 08	2.92*E* − 07	1.86*E* − 07	2.05*E* − 07	1.84*E* − 08	4.54*E* − 06	5.17*E* − 05
0.4	1.70*E* − 08	4.36*E* − 08	8.23*E* − 07	3.25*E* − 08	5.91*E* − 08	2.60*E* − 07	1.45*E* − 07	9.79*E* − 07	9.90*E* − 07	6.50*E* − 07	2.85*E* − 06	1.40*E* − 05
0.5	2.05*E* − 08	2.92*E* − 08	2.55*E* − 07	1.18*E* − 08	4.18*E* − 08	2.53*E* − 07	2.21*E* − 07	6.61*E* − 07	2.39*E* − 07	1.95*E* − 07	3.33*E* − 06	2.99*E* − 05
0.6	8.47*E* − 09	1.09*E* − 07	2.52*E* − 08	2.84*E* − 08	4.07*E* − 08	2.80*E* − 07	3.06*E* − 07	7.81*E* − 07	6.40*E* − 07	7.70*E* − 08	2.20*E* − 06	1.64*E* − 06
0.7	2.48*E* − 08	1.39*E* − 07	6.13*E* − 07	4.73*E* − 08	7.41*E* − 08	3.00*E* − 07	3.41*E* − 07	6.71*E* − 07	8.51*E* − 07	4.43*E* − 07	1.92*E* − 06	1.98*E* − 05
0.8	4.69*E* − 08	1.99*E* − 07	4.12*E* − 07	8.42*E* − 08	2.53*E* − 08	2.41*E* − 07	3.16*E* − 07	6.54*E* − 08	3.21*E* − 07	3.47*E* − 08	4.15*E* − 06	2.21*E* − 05
0.9	7.91*E* − 08	4.48*E* − 07	1.05*E* − 06	1.97*E* − 07	8.91*E* − 08	7.07*E* − 07	7.50*E* − 07	1.05*E* − 06	2.81*E* − 06	2.20*E* − 07	1.61*E* − 05	5.19*E* − 05
1.0	1.04*E* − 06	2.26*E* − 06	5.54*E* − 06	1.37*E* − 06	1.07*E* − 06	3.76*E* − 06	3.59*E* − 06	5.05*E* − 06	9.58*E* − 04	1.09*E* − 03	1.05*E* − 03	2.39*E* − 03

**Table 5:** Statistical analysis of the results for MAD, ENSE, RMSE, and NSE obtained by multiple executions of the NARX-BLM algorithm for the condensation film problem with Pr=*δ*=1.

	MAD			ENSE			RMSE			TIC			NSE		
	Min	Mean	Std	Min	Mean	Std	Min	Mean	Std	Min	Mean	Std	Min	Mean	Std
Θ(*η*)	5.45*E* − 06	8.51*E* − 06	5.30*E* − 06	1.98*E* − 12	6.06*E* − 12	7.08*E* − 12	7.26*E* − 06	7.78*E* − 06	9.03*E* − 07	1.54*E* − 06	1.65*E* − 06	1.92*E* − 07	1	1	7.08*E* − 12
Ψ(*η*)	5.81*E* − 06	8.65*E* − 06	3.59*E* − 06	5.55*E* − 16	1.30*E* − 15	1.01*E* − 15	4.03*E* − 06	5.29*E* − 06	1.57*E* − 06	1.32*E* − 08	1.73*E* − 08	5.11*E* − 09	1	1	5.77*E* − 16
*k*(*η*)	2.04*E* − 05	3.60*E* − 05	1.69*E* − 05	9.19*E* − 13	3.30*E* − 12	2.84*E* − 12	3.11*E* − 05	3.86*E* − 05	1.13*E* − 05	1.21*E* − 06	1.51*E* − 06	4.43*E* − 07	1	1	2.84*E* − 12
−*s*(*η*)	1.47*E* − 05	3.83*E* − 05	2.51*E* − 05	4.16*E* − 13	3.61*E* − 12	3.93*E* − 12	2.27*E* − 05	3.09*E* − 05	7.48*E* − 06	8.23*E* − 07	1.12*E* − 06	2.71*E* − 07	1	1	3.93*E* − 12
*θ*(*η*)	1.00*E* − 05	2.49*E* − 04	2.46*E* − 04	8.38*E* − 13	7.23*E* − 12	8.64*E* − 12	2.51*E* − 04	4.53*E* − 04	2.58*E* − 04	8.06*E* − 07	1.45*E* − 06	8.27*E* − 07	1	1	8.64*E* − 12

**Table 6:** Results of performance function in terms of mean square error (MSE) and gradient values with different activation functions for condensation film problem with Pr=10 and *δ*=1.0.

	Log-sigmoid				Tan-hyperbolic			
	Mean square error		Gradient		Mean square error		Gradient	
	*n* = 60	*n* = 30	*n* = 60	*n* = 30	*n* = 60	*n* = 30	*n* = 60	*n* = 30
Θ	5.92*E* − 15	9.32*E* − 14	8.43*E* − 11	2.53*E* − 09	2.14*E* − 12	1.50*E* − 11	5.18*E* − 10	5.24*E* − 10
Ψ	1.35*E* − 14	6.03*E* − 14	5.19*E* − 11	5.03*E* − 11	8.44*E* − 13	1.39*E* − 14	1.77*E* − 10	6.64*E* − 11
*k*	6.58*E* − 12	3.83*E* − 12	6.40*E* − 11	5.20*E* − 08	3.66*E* − 12	1.94*E* − 10	4.12*E* − 09	9.02*E* − 10
−*s*	2.57*E* − 13	1.48*E* − 10	1.03*E* − 10	3.47*E* − 11	3.40*E* − 12	1.85*E* − 10	7.69*E* − 10	6.28*E* − 11
*θ*	1.34*E* − 10	6.35*E* − 09	2.46*E* − 10	8.92*E* − 09	1.04*E* − 08	1.04*E* − 08	8.93*E* − 09	9.15*E* − 09

The article "Investigation of Three-Dimensional Condensation Film Problem over an Inclined Rotating Disk Using a Nonlinear Autoregressive Exogenous Model" was published in 2022. Journal: Comput Intell Neurosci.

## Data Availability

The data that support the findings of this study are available from the corresponding author upon reasonable request.
